This article has been retracted.

# Nomogram-Based Prediction of Overall and Cancer-Specific Survival in Patients with Primary Bone Diffuse Large B-Cell Lymphoma: A Population-Based Study

**DOI:** 10.1155/2022/1566441

**Published:** 2022-05-05

**Authors:** Xing-yao Yang, Xin He, Yun Zhao

**Affiliations:** Department of Orthopaedics, The Fifth People's Hospital of Chengdu, Sichuan 611130, China

## Abstract

**Background:**

Primary bone diffuse large B-cell lymphoma (PD-DLBCL) accounts for more than 80% of primary bone lymphoma. We created two nomograms to predict overall survival (OS) and cancer-specific survival (CSS) in patients with PD-DLBCL for this rare disease.

**Methods:**

In total, 891 patients diagnosed with PB-DLBCL between 2007 and 2016 were extracted from the Surveillance, Epidemiology, and End Results (SEER) database. Univariate and multivariate Cox analyses were performed to explore independent prognostic factors and create nomograms for OS and CSS. The area under the curve (AUC), the calibration curve, decision curve analysis (DCA), and Kaplan–Meier (K-M) curve analysis were used to evaluate the nomograms.

**Results:**

Four variables were identified as independent prognostic factors for OS, and three variables were identified as independent prognostic factors for CSS. The receiver operating characteristic (ROC) curves demonstrated the strong discriminatory power of the nomograms. The calibration and DCA curves showed that the nomograms had a satisfactory ability to predict OS and CSS. The K-M curves showed that age, gender, primary site, chemotherapy, and tumor stage affected patient survival.

**Conclusions:**

In patients with PD-DLBCL, age, race, primary site, and chemotherapy affected OS, while age, race, and chemotherapy affected CSS. The two nomograms created based on the aforementioned variables provided more accurate individual survival predictions for PD-DLBCL patients and can help physicians make appropriate clinical decisions.

## 1. Background

A preprint has previously been published [1]. Primary bone lymphoma (PBL) was called primary reticulocyte sarcoma by Oberlin in 1928 and precisely defined by Shoji et al. in 1971 [2]. With the advancement of medical technology, PBL has been recognized as a malignant tumor of bone originating from the hematopoietic system. It is also a rare form of extranodal lymphoma and also accounts for 3%–7% of extranodal lymphomas [3]. The disease has no specific manifestations in its early stages; the first symptoms are fever, the appearance of lumps, and weight loss [4]. PBL can occur in all bones of the body but is most common in the femur and the pelvis [5]. The age of onset is typically 45–60 years old. Men are slightly more likely to develop the disease than women; this trend seems to have increased in recent years, though the factors leading to its occurrence are less clear [6].

More than 80% of the pathological types of PBL are primary bone diffuse large B-cell lymphoma (PD-DLBCL) [3, 7]. Due to PD-DLBCL heterogeneity, there is no standard treatment plan. The treatment options are chemotherapy, radiotherapy, and surgery. Surgery is only used for symptoms of compression, pathological fractures, or biopsies. Currently, CHOP and CHOP-like regimens are commonly used for chemotherapy. Bruno Ventre et al. [4] showed that anthracycline-based regimens were more effective and that PD-DLBCL patients treated with chemotherapy were significantly better than those treated with radiotherapy.

The effectiveness of radiotherapy as a consolidation modality after chemotherapy is controversial [8, 9]. Held et al. [10] showed that radiotherapy helped improve PB-DLBCL patient survival. However, many factors affect the survival rate of PB-DLBCL patients, and, to our knowledge, no study to date has predicted or analyzed the relationship between clinical characteristics and survival among PB-DLBCL patients. To address this gap, we used the Surveillance, Epidemiology, and End Results (SEER) program database to predict survival and analyze the clinical characteristics of patients with PB-DLBCL.

## 2. Method

### 2.1. Patients

The SEER database contains epidemiological information from 18 cancer registries in the United States (US). Most importantly, it is a publicly available database covering 30% of the entire US population, reducing ethical conflicts by an overwhelming extent. We applied the following inclusion criteria to SEER Stat (8.3.9.2) data from 2007 to 2016: (1) confirmed PB-DLBCL histological type (histological code 9680/3 in the third edition of the International Album of Oncological Diseases); (2) primary tumor; (3) bone only (position code C40.0-C41.9 in the third edition of the International Album of Oncological Diseases); and (4) follow-up information completed. We applied the following exclusion criteria: (1) incomplete information on age, gender, race, pathological type, radiotherapy, chemotherapy, and/or tumor metastasis; (2) survival time <1 month; and (3) nonbone disease onset. The 891 patients who met the inclusion criteria were randomly divided into a training set (70%) and a test set (30%).

We built nomograms using the training cohort and validated them using the validation cohort. Then, we analyzed the overall survival (OS) and cancer-specific survival (CSS) of patients.

### 2.2. Data Analysis

We examined the following variables: age, race, gender, primary site, surgery, radiotherapy, chemotherapy, and tumor stage (localized, regional, distant). We used X-tile software (Yale University, New Haven, CT, USA) to better determine the cutoff value of the continuous variable of age. The training cohort was screened for the variables using the univariate Cox regression model (*P* < 0.2). The screened variables were enrolled in multivariate Cox regression to clarify the independent risk factors for OS and CSS in PB-DLBCL patients (*P* < 0.05), which were then plotted in the nomograms. The effect of the independent risk factors on OS and CSS in PB-DLBCL patients was demonstrated using K-M curves and log-rank tests. ROC and calibration curves were used to confirm the accuracy of the nomogram. A decision curve analysis (DCA) curve was used to calculate the net benefit in order to determine the predictive effect of the nomogram on the clinical outcomes. All data were analyzed using the statistical software R (version 3.43, https://www.r-project.org).

## 3. Results

### 3.1. Demographic Characteristics

We collected SEER database information from 2007 to 2016 for 891 patients with PB-DLBCL (Table 1). The data were divided into a training cohort (*N* = 627) and a validation cohort (*N* = 264). In total, there were 500 (56.1%) male and 391 (43.9%) female patients in the sample. The primary tumors were located in the mandible, skull, pelvis, spine, ribs, and other axial sites in 560 patients (62.9%) and in the extremities in 331 patients (37.1%). Regarding treatment, 154 (17.3%) PB-DLBCL patients received surgery, 488 (54.8%) received radiotherapy, and 776 (87.1%) received chemotherapy. Most patients were in the localized stage (461, 51.7%), 129 (14.5%) were in the regional stage, and 301 (33.8%) were in the distant stage.

### 3.2. Variable Screening and Nomogram Creation

First, we used X-tile software to determine the optimal cutoff for age, dividing age into 7–62 years old, 63–75 years old, and >75 years old (Figure 1). Before creating the nomograms, we performed univariate and multivariate regression analyses for age, race, gender, primary site, surgery, chemotherapy, radiotherapy, and tumor stage. The univariate analysis for OS suggested that age, race, gender, primary site, and chemotherapy were independent risk factors. However, in the subsequent multivariate analysis, gender was not found to be an independent risk factor (Table 2). Regarding CSS, age, race, gender, primary site, chemotherapy, and tumor stage were considered independent risk factors in the univariate analysis, while only age, race, and chemotherapy information were considered independent risk factors in the multivariate analysis (Table 3).

The variables were used to construct a nomogram, and patient prognosis was predicted by calculating the total score (Figure 2). Subsequently, the accuracy of the nomogram was verified. The ROC curve showed that the nomogram had a better discrimination ability (Figure 3). In addition, the calibration curve effectively demonstrated the accuracy of the nomogram prediction versus the actual probability of survival (Figure 4). The DCA curve confirmed that the nomogram had net benefit and could effectively improve patient outcomes (Figure 5).

### 3.3. Risk Factor Analysis

Patient survival was assessed using K-M curves. As shown, longer OS was associated with younger age (*P* < 0.001), male gender (*P*=0.024), primary site in the extremities (*P* < 0.001), chemotherapy treatment (*P* < 0.001), and regional tumor stage (*P*=0.05). Race (*P* =0.65), whether or not the patient had surgery (*P*=0.25), and radiotherapy treatment (*P*=0.75) did not have a significant effect on OS (Figure 6).

## 4. Discussion

As an independent and rare disease, PB-DLBCL research has been limited to case reports and small-sample retrospective studies. However, it is crucial to summarize the pathological features of PB-DLBCL, effectively predict the prognosis, and deepen physicians' understanding of the disease. A nomogram is a statistical tool that can integrate multiple prognostic risk factors in the clinic, neutralize various patient factors, incorporate them into a prognostic evaluation, and display them visually [11]. The correct use of nomograms can improve patient outcomes and assist clinicians in making accurate survival assessments and treatment decisions [12].

In the present study, based on the SEER database, we used the Cox proportional hazards model to screen out risk factors, constructed nomograms, and then used the K-M curve to evaluate the survival of patients. The good predictive and clinical net benefits of the nomogram were demonstrated by the ROC, calibration, and DCA curves. As far as we know, this is the first study to construct a nomogram for PB-DLBCL and analyze prognostic factors.

Using Cox multivariate analysis, we learned that age, race, gender, primary site, chemotherapy, and tumor stage were risk factors associated with survival. In addition, the nomogram showed that PB-DLBCL is a disease with a good prognosis. Furthermore, although PB-DLBCL is highly malignant, even some elderly people can survive for a long time after diagnosis [13]. This finding is in line with the results of some previous studies in which the PB-DLBCL five-year survival rate exceeded 70% [4, 14].

Some retrospective studies with small samples found a higher incidence rate among males than females [15, 16]. Likewise, using the K-M curves, we found that OS was higher in men than in women. Age has always been an important factor affecting many malignancies. For example, Wang et al. [7] found that patients with malignant PBL had a higher risk of death from OS and CSS in patients over 61 years old, risk of death up to 7 times. Although our findings also showed that older patients have a higher risk of death for OS and CSS, this question should be analyzed comprehensively, as many older patients have a poor physical condition, which contributes to increased mortality. The same is true for race. Due to the limitations of the SEER database, the majority of patients in our sample population were white, which may have caused data bias.

PB-DLBCL can occur in all bones of the body, with long bones and the spine being the most common [17]. Upon imaging, approximately 70% showed osteolytic destruction [18]. In the present study, we found that the primary site of the tumor affected patient's OS and CSS. Survival was significantly lower for tumors in the spine than in the extremity bones. This phenomenon may be related to the compression of nerves by spinal lesions, which can lead to more severe complications, such as paralysis and reduced survival [19].

In recent years, many studies have been conducted on the best treatment options for PB-DLBCL. CHOP and CHOP-like regimens are commonly used for chemotherapy; however, there are no clear guidelines for combination regimens. Bruno Ventre et al. [4] found a good prognosis for patients with PB-DLBCL who received anthracycline-based chemotherapy regimens with or without the administration of radiotherapy regimens. However, for patients receiving radiotherapy, the use of larger radiation fields and doses was not associated with better outcomes. Meanwhile, Pfreundschuh et al. [19] suggested that rituximab in combination with CHOP-like chemotherapy regimens improves the long-term prognosis of young patients with PB-DLBCL. Bhagavathi and Fu's study [20] found that the addition of rituximab increased three-year progression-free survival (PFS) from 52% to 88%. Radiotherapy used the usual doses for non-Hodgkin's lymphoma (35–45 Gy in 1.8–2 Gy fractions) [21]. Numerous scholarly studies have suggested that radiotherapy should only be used for treatment as a consolidation option [9]. Furthermore, in the present study, the surgical treatment factor did not affect patient survival. Some studies have also mentioned that surgery does not seem to be a necessary option for patients with PB-DLBCL [13, 22]. With the progress of chemotherapy and radiotherapy, most surgical operations have been used to clarify the nature of lesions.

Of course, there are some limitations to the present study. First, we only used the SEER database and did not use information from other databases for external validation. In addition, the SEER database lacks some important information, such as disease progression, comorbidities, and complications, as well as specific information on radiotherapy and chemotherapy. We plan to address this lack of information in future research. However, these issues did not affect the results obtained in the present study. Although these factors made the study imperfect, we were able to evaluate the impact of various factors on the survival of patients with PB-DLBCL, and the line graphs can help clinicians predict the prognosis of their patients.

## 5. Conclusion

The current study identified age, race, primary site, and chemotherapy as variables affecting OS in PD-DLBCL patients and age, race, and chemotherapy as variables affecting CSS. These factors were incorporated into the construction of the nomograms, which provided more accurate individual survival predictions for PD-DLBCL patients to some extent in order to help physicians make appropriate clinical decisions.

## Figures and Tables

**Figure 1:** Optimal cutoff age based on X-tile analysis. (a) The black spot indicates that the optimal cutoff age has been determined. (b) Histograms and (c) Kaplan–Meier curves were constructed based on the determined cutoff values.

**Figure 2:** Nomograms predicting three- and five-year OS and CSS in patients with PB-DLBCL. OS = overall survival; CSS = cancer-specific survival; PB-DLBCL = primary bone diffuse large B-cell lymphoma.

**Figure 3:** ROC curves predicting three- and five-year OS and CSS in PB-DLBCL patients. (a) ROC curves for three- and five-year OS for the training cohort. (b) ROC curves for three- and five-year CSS for the training cohort. (c) ROC curves for three- and five-year OS for the validation cohort. (d) ROC curves for three- and five-year CSS for the validation cohort. OS = overall survival; CSS = cancer-specific survival; PB-DLBCL = primary bone diffuse large B-cell lymphoma.

**Figure 4:** Calibration curves predicting three- and five-year OS and CSS in patients with PB-DLBCL. (a) Calibration curves for three- and five-year OS for the training cohort. (b) Calibration curves for three- and five-year OS for the validation cohort. (c) Calibration curves for three- and five-year CSS for the training cohort. (d) Calibration curves for three- and five-year CSS for the validation cohort. OS = overall survival; CSS = cancer-specific survival; PB-DLBCL = primary bone diffuse large B-cell lymphoma.

**Figure 5:** Nomograms of decision curve analysis, (a) (OS, five years) and (b) (CSS, five years). The *x*-axis represents the threshold probability, and the *y*-axis represents the net benefit.

**Figure 6:** Survival curves for factors associated with healing in 891 patients.

**Table 1:** Patient demographic characteristics.

	Training cohort *N* (%)	Validation cohort *N* (%)	Total *N* (%)
*N*	627	264	891
Age (%)			
7–62 years old	340 (54.2)	142 (53.8)	482 (54.1)
63–75 years old	160 (25.5)	71 (26.9)	231 (25.9)
>75 years old	127 (20.3)	51 (19.3)	178 (20.0)
Race (%)			
White	536 (85.5)	228 (86.4)	764 (85.7)
Black	43 (6.9)	18 (6.8)	61 (6.8)
Others	48 (7.7)	18 (6.8)	66 (7.4)
Gender (%)			
Male	342 (54.5)	158 (59.8)	500 (56.1)
Female	285 (45.5)	106 (40.2)	391 (43.9)
Primary site (%)			
Axial	404 (64.4)	156 (59.1)	560 (62.9)
Appendix	223 (35.6)	108 (40.9)	331 (37.1)
Surgery (%)			
Yes	104 (16.6)	50 (18.9)	154 (17.3)
No	523 (83.4)	214 (81.1)	737 (82.7)
Radiation (%)			
Yes	342 (54.5)	146 (55.3)	488 (54.8)
No	285 (45.5)	118 (44.7)	403 (45.2)
Chemotherapy (%)			
Yes	543 (86.6)	233 (88.3)	776 (87.1)
No	84 (13.4)	31 (11.7)	115 (12.9)
Stage (%)			
Localized	314 (50.1)	147 (55.7)	461 (51.7)
Regional	92 (14.7)	37 (14.0)	129 (14.5)
Distant	221 (35.2)	80 (30.3)	301 (33.8)

**Table 2:** Univariate and multivariate analysis of OS in the training cohort.

Characteristics	Univariate analysis HR (95% CI)	*P* value	Multivariate analysis HR (95% CI)	*P* value
Age	3.2 (2.61–3.91)	0	2.97 (2.4–3.66)	0
7–62 years old				
63–75 years old				
>75 years old				
Race	1.19 (0.92–1.53)	0.179	1.25 (0.98–1.59)	0.0726
White				
Black				
Others				
Gender	1.35 (0.98–1.85)	0.066	0.88 (0.64–1.22)	0.4513
Male				
Female				
Primary site	0.53 (0.36–0.76)	0.001	0.67 (0.46–0.97)	0.0337
Axial				
Appendix				
Surgery	1.07 (0.69–1.64)	0.772	NA	NA
Yes				
No				
Radiation	0.85 (0.62–1.18)	0.339	NA	NA
Yes				
No				
Chemotherapy	4.05 (2.88–5.7)	0	3.08 (2.17–4.37)	0
Yes				
No				
Stage	1.09 (0.92–1.3)	0.321	NA	NA
Localized				
Regional				
Distant				

**Table 3:** Univariate and multivariate analysis of CSS in the training cohort.

Characteristics	Univariate analysis HR (95% CI)	*P* value	Multivariate analysis HR (95% CI)	*P* value
Age	3.14 (2.13–4.63)	0	2.56 (1.68–3.9)	0
7–62 years old				
63–75 years old				
>75 years old				
Race	5.57 (2.92–10.66)	0	4.44 (2.08–9.48)	0.001
White				
Black				
Others				
Gender	1.7 (0.92–3.14)	0.089	1.1 (0.56–2.17)	0.7749
Male				
Female				
Primary site	0.43 (0.21–0.87)	0.019	0.71 (0.33–1.5)	0.3701
Axial				
Appendix				
Surgery	0.71 (0.34–1.47)	0.36	NA	NA
Yes				
No				
Radiation	0.67 (0.35–1.27)	0.219	NA	NA
Yes				
No				
Chemotherapy	1.35 (0.97–1.87)	0.079	1.63 (1.11–2.39)	0.0128
Yes				
No				
Stage	2.28 (0.81–6.39)	0.118	2.28 (0.78–6.69)	0.1338
Localized				
Regional				
Distant				

## Data Availability

Our data are available from the Surveillance, Epidemiology, and End Results (SEER) research database. This is a public research database.
